# Clinical Efficacy of Bendamustine Plus Rituximab (BR) for B-cell Relevant Indolent Non-Hodgkin's Lymphoma and Role of *β*2-MG in Predicting the Efficacy of BR Regimen: A Real-World Retrospective Study in China

**DOI:** 10.1155/2022/1080879

**Published:** 2022-01-20

**Authors:** Yujie Zhang, Donghua He, Jingsong He, Weijia Huang, Yang Yang, Zhen Cai, Yi Zhao

**Affiliations:** Bone Marrow Transplantation Center, The First Affiliated Hospital, Zhejiang University School of Medicine, Hangzhou City, Zhejiang Province, 310003, China

## Abstract

**Background:**

Domestic bendamustine has been approved for appearing on the market in China in the past two years. The report on bendamustine plus rituximab (BR) in the treatment of Chinese B-cell-associated indolent non-Hodgkin's lymphoma (iNHL) has not yet been published. This study probed into clinical efficacy of the BR regimen for B-cell-associated iNHL in China as well as the value of *β*2-microglobulin (*β*2-MG) as a prognostic factor.

**Methods:**

We retrospectively analyzed clinical data of 73 B-cell-associated iNHL patients who received BR treatment in The First Affiliated Hospital, College of Medicine, Zhejiang University from January 2020 to January 2021, including clinical characteristics, therapies, therapeutic efficacy, and prognosis-related factors. Thirty-three patients (45.2%) did not receive any other treatment before the BR regimen, and other patients received CHOP, R-CHOP, and other regimens in the past. The cutoff date for follow-up was May 2021. Clinical characteristics of patients were analyzed. The clinical efficacy of the BR regimen was evaluated. Differences of *β*2-MG expression before and after treatment were analyzed between the CR+PR group and the SD+PD group. Main outcomes were progression-free survival (PFS) and overall survival (OS). A multivariate Cox regression model was taken to analyze prognostic factors relative to survival rate of patients, and adverse events (AEs) during treatment.

**Results:**

The objective response rate (ORR) of B-cell-associated iNHL patients who received BR regimen as first-/multiline treatment was 79.5%, with complete response (CR) of 37.0%, partial response (PR) of 42.5%, median PFS of 12.1 months (95% confidence interval (CI): 10.9-13.2), and median OS of 15.5 months (95% CI: 14.8-16.1). Before treatment, there was no statistical significance in the *β*2-MG level between the CR+PR group and the SD+PD group (*p* > 0.05). After treatment, the *β*2-MG level in the CR group was noticeably lower than that in the SD+PD group (*p* < 0.05). The *β*2-MG level in the CR+PR group decreased conspicuously after treatment (*p* < 0.05). The *β*2-MG level in the SD+PD group after treatment was not notably different from that before treatment (*p* > 0.05). According to the median expression level of *β*2-MG before treatment, patients were divided into two groups. The average PFS of the low expression group was 12.69 ± 0.77 months, which was longer than the high expression group (10.13 ± 0.74 months), but the difference between the groups was not statistically significant (*p* > 0.05). Multivariate Cox regression analysis showed that B-cell-associated iNHL subtype was the independent prognostic marker most likely to affect PFS of patients (*p* = 0.051). Incidence of any grade of AEs in all patients was 32.9% (24/73).

**Conclusion:**

B-cell-associated iNHL patients who received BR regimen had favorable clinical efficacy and were tolerable to AEs. Though the *β*2-MG level in this study could not be used to predict clinical outcome, a lower level before treatment seemed to be implicated in better survival outcomes of patients. Our research also unraveled that B-cell-associated iNHL subtype may be a key factor to patient's prognosis. Overall, this study offers some important insights into clinical application of the BR regimen for Chinese B-cell-associated iNHL patients.

## 1. Introduction

Lymphoma is one of the top 10 cancers in the world, including Hodgkin's lymphoma (HL) and non-Hodgkin's lymphoma (NHL). The year 2017 witnessed 488,000 NHL cases and 249,000 NHL-related deaths worldwide [1]. NHL deriving from B-cells can be classified into B-cell-associated indolent NHL (iNHL) and B cell-associated invasive NHL in line with its invasiveness [2]. B-cell-associated iNHL includes follicular lymphoma (FL), lymphoplasmacytic lymphoma (LPL), marginal zone lymphoma (MZL), indolent mantle-cell lymphoma, Waldenstrom's macroglobulinemia, and chronic lymphocytic leukemia (CLL) [3]. These patients have relatively favorable survival outcomes, whereas advanced B-cell-associated iNHL is still considered incurable, which is called the iNHL paradox [2, 4]. In China, rituximab plus cyclophosphamide, doxorubicin, vincristine, and prednisone (R-CHOP) regimen is generally taken as a first-line regimen for B-cell-associated iNHL treatment, but in western countries, bendamustine plus rituximab (BR) regimen has been approved for the first-line treatment of iNHL for many years [3, 5, 6]. Owing to poor outcomes of patients being refractory to the R-CHOP regimen, researchers engage in seeking novel treatment regimens.

Bendamustine as a novel alkylating agent has been approved for the treatment of iNHL including CLL [7–9]. The introduction of rituximab is believed to improve survival outcomes of FL patients [4]. Regimens containing rituximab have also been affirmed in the management of elderly patients with B-cell-associated iNHL [10]. Several randomized trials have demonstrated that the BR regimen can improve progression-free survival (PFS) compared with the R-CHOP regimen [11–13]. Indeed, data from several clinical trials have shown that the overall response rate ranges from 69 to 93% with the BR regimen [11, 14, 15]. Domestic bendamustine has been approved for appearing on the market in China in the past two years. The report on BR in the treatment of Chinese B-cell-associated indolent non-Hodgkin's lymphoma (iNHL) has not yet been published. Besides, the prognostic value of *β*2-microglobulin (*β*2-MG) in patients with NHL was evaluated previously. Kanemasa et al. [16] authenticated that *β*2-MG level is a key prognosticator for patients with diffuse large B-cell lymphoma (DLBCL), but its clinical and prognostic significance in B-cell-associated iNHL remains to be elucidated.

To this end, we carried out a retrospective study on real-world data from the Chinese cohort and made a thorough inquiry into the clinical efficacy of BR regimen for B-cell-associated iNHL as well as the value of *β*2-MG as a prognostic factor. Most clinical research regarding the BR regimen for iNHL is conducted in Western countries. Nevertheless, there is less clinical experience in China. Our investigation may be available for clinical practice of the BR regimen in China.

## 2. Materials and Methods

### 2.1. Participants

A retrospective analysis was carried out on clinical data from 73 patients with B-cell-associated iNHL who received BR regimen in The First Affiliated Hospital, College of Medicine, Zhejiang University from January 2020 to January 2021. After admission, all patients required a bone marrow biopsy, ultrasound of superficial lymph nodes, and positron emission tomography-computed tomography (PET-CT) or enhanced CT scan. All patients were diagnosed by histopathological assessment and immunohistochemical study consistent with the 2016 Revision of the World Health Organization Classification of Lymphoid Neoplasms [17]. Classification of most types of lymphoma refers to the Lugano classification (2014) [18]. In addition, a method proposed by Rai et al. [19] or Binet et al. [20] was adopted for CLL classification. All collected patients met the following criteria: all patients were ≥18 years old; International Prognostic Index (IPI) was 1-5. The main exclusion criteria were as follows: patients who were intolerant to BR and then switched to other regimens; patients who had central nervous system lymphoma or primary mediastinal large B-cell lymphoma (PMBCL), with clear evidence of uncontrolled concomitant diseases. This study was approved by the Medical Ethics Committee of The First Affiliated Hospital, College of Medicine, Zhejiang University following the guidelines of the international coordination meeting (Good Clinical Practice; The Declaration of Helsinki).

### 2.2. Procedures

All patients received BR regimen as follows: 375 mg/m^2^ rituximab (NMPN J20170034; Roche Pharma Ltd.), d1 of each cycle, administrated as an intravenous infusion (specification: 100 mg/10 mL), for 6 cycles (4 weeks a cycle); 75 mg/m^2^ bendamustine (national medicine permission number (NMPN) H20193358; Chia Tai Tianqing Pharmaceutical Group Co., Ltd.), d2~d3 of each cycle, administrated as an intravenous infusion (specification: 25 mg), for 6 cycles (4 weeks a cycle). Regimens were changed following clinical needs when the lymph node regression was found to be less than 50% or there was evidence of disease progression before the entire treatment plan was completed.

### 2.3. Therapeutic Evaluation

One day before treatment and one week after treatment, 5 mL fasting venous blood was collected from each subject in the morning, centrifuged to separate the serum, stored, and prepared at -80°C. The Automatic Hitachi 7080 Biochemistry Analyzer was implemented to assess serum *β*2-MG level.

Based on Cheson's revised response criteria [21], treatment response was categorized as CR, partial response (PR), stable disease (SD), and progressive disease (PD). The primary efficacy endpoint was CR assessed by PET and Independent Review Committee (IRC) per Lugano classification (2014) [18]. Other outcomes included objective response rate (ORR), progression-free survival (PFS), and overall survival (OS). Safety endpoints involved the incidence of all grades of adverse events (AEs).

### 2.4. Follow-Up Visit

Special personnel was in charge of following up all the patients through telephone, WeChat, QQ, and other communication methods. The follow-up visit was stopped in May 2021. PFS and OS of patients were recorded (PFS: the time from the start of treatment to disease relapse or progression; OS: the time from the start of treatment to death or loss of follow-up).

### 2.5. Statistical Analysis

All statistical analyses were done using SPSS software (version 25.0; SPSS, Chicago, Illinois). Categorical variables were expressed as the number of cases and percentages. The chi-square test or Fisher's exact test was used for comparison between two categorical variables. Kolmogorov-Smirnov statistics were implemented to test the assumption of normality of continuous variables. If the data were normally or close to normally distributed, they were expressed as the mean (M) ± standard deviation (SD). The independent-samples *t*-test compared scores on the same variable but for two different groups of cases. While the paired *t*-test compared scores on two different variables but for the same group of cases. Otherwise, the data were expressed as IQR. The Mann–Whitney *U* test was taken to compare the differences between two different groups. The Kaplan-Meier method was utilized to assess PFS and OS. The log-rank test was employed for PFS and OS comparison between two groups. Multivariate Cox regression analysis was handled to measure variables of dismal prognosis. *p* < 0.05 was considered statistically significant.

## 3. Results

### 3.1. Baseline Characteristics of Patients

Among 73 patients, 40 (54.8%) patients received other therapeutic regimens previously. The common subtypes were follicular lymphoma (27.4%) (20/73), mantle cell lymphoma (23.3%) (17/73), mucosa-associated lymphoid tissue (24.7%, 18/73), and lymphocytic lymphoma (15.1%, 11/73). The median age of all patients was 62 (56–69). Baseline characteristics of patients are listed in Table 1.

### 3.2. Clinical Efficacy

ORR of patients who received BR regimen was 79.5%, with CR of 37.0% and PR of 42.5%. Median PFS was 12.1 months (95% confidence interval (CI): 10.9-13.2) (Table 2). Median OS was 15.5 months (95% CI: 14.8-16.1). Survival curves are illustrated in Figure 1.

### 3.3. Changes of *β*2-MG Level during Treatment

Patients were classified into the CR+PR group and SD+PD patient according to whether patients achieved CR+PR. The independent samples *t*-test compared the *β*2-MG level between the CR+PR group and the SD+PD group (CR+PR before treatment vs. SD+PD before treatment; CR+PR after treatment vs. SD+PD after treatment). As illustrated in Figure 2, there was no significant difference in the *β*2-MG level between the CR+PR group and the SD+PD group before treatment (*p* > 0.05). While after treatment, the *β*2-MG level in the CR+PR group was lower than that in the SD+PD group (*p* < 0.05). Afterward, paired *t*-tests compared *β*2-MG level changes in the same group (CR+PR before treatment vs. CR+PR after treatment; SD+PD before treatment vs. SD+PD after treatment). As shown in Figure 3, the *β*2-MG level in the CR+PR group was decreased conspicuously after treatment (*p* < 0.05), and that in the SD+PD group was downregulated after treatment, but the difference was not statistically significant (*p* > 0.05).

### 3.4. Correlation between *β*2-MG and Survival Outcome

We investigated the correlation between *β*2-MG expression level before treatment/after treatment/the change rate before and after treatment and the survival outcomes of patients.

Patients were classified into the *β*2‐MG < 3.25 mg/L group and the *β*2‐MG ≥ 3.25 mg/L group following the median *β*2-MG expression level before treatment. The survival analysis of PFS and OS depicted that the difference between two groups was not statistically significant (PFS: *p* > 0.05; OS: *p* > 0.05) (Figure 4). Following the median *β*2-MG expression level after treatment, patients were grouped into the *β*2‐MG < 2.77 mg/L group and the *β*2‐MG ≥ 2.77 mg/L group. The survival analysis of PFS and OS disclosed that the difference between two groups was not statistically significant (PFS: *p* > 0.05; OS: *p* > 0.05) (Figure 5). Following the change rate of *β*2-MG expression level before and after treatment (Figure 6), patients were sorted into the change rate < 0 group and the change rate > 0 group. PFS and OS survival analysis denoted that there was no significant difference between two groups (PFS: *p* > 0.05; OS: *p* > 0.05).

In addition, multivariate Cox regression analysis was carried out according to sex, age, indolent B-cell lymphoma subtype, stage, ECOG PS, number of previous lines of therapy, and *β*2-MG level. As detailed in Table 3, indolent B-cell lymphoma subtype was the independent prognostic marker most likely to affect PFS of patients.

### 3.5. AEs

The incidence of any grade of AEs in all patients was 32.9% (24/73). Most patients suffered multiple AEs, and these symptoms improved after corresponding treatment. Among them, leukopenia (6 cases), pulmonary infections (4 cases), fever (3 cases), fatigue (4 cases), nausea and emesis (3 cases), and skin rash (1 case) are the major AEs (Table 4). After reverification, there were 5 cases of severe hematological AEs (grade 3-4), 1 case of obvious nausea and emesis. The incidence of serious AEs was 8.2% (6/73). No patients stopped medication or adjusted dose due to adverse drug reactions during this period.

## 4. Discussion

Aggressive and indolent lymphomas are the two subtypes of B-cell-derived NHL, which are usually treated with different regimens. We retrospectively analyzed the clinical outcomes of 73 patients with B-cell-associated iNHL. It was unraveled that the BR regimen had good efficacy and safety in B-cell-associated iNHL patients. Besides, we investigated the clinical significance of *β*2-MG in B-cell-associated iNHL. Unfortunately, based on research samples in this study, *β*2-MG does not seem to be able to guide these patients to receive the prognosis after the BR regimen, which may be caused by small sample size, because the BR regimen has just been applied in clinical practice in China not long ago.

At present in China, the R-CHOP regimen remains a standard therapy for most NHL patients, including B-cell-associated iNHL. In the BRIGHT study [13], clinical efficacy and safety of the R-CHOP/R-CVP or BR regimen in the first-line treatment of B-cell-associated iNHL were compared, and the efficacy of the BR regimen for the long-term clinical benefit of patients was proved. Both bendamustine and cyclophosphamide belong to alkylating agents, but some scholars believed that bendamustine can repress mitotic checkpoint protein to interrupt or stop cell division of cancer cells [22]. Further clarification of the pharmacological mechanism of bendamustine in antitumor may unveil differences in clinical benefits between R-CHOP and BR regimens in the management of B-cell-associated iNHL. A prospective, multicenter, open-label, single-arm, phase 3 study demonstrated the efficacy and safety of bendamustine in Chinese adults with indolent B-cell NHL who relapsed after chemotherapy and rituximab treatment, with results similar to those of previous clinical trials conducted in patients from Western countries [23], which seems to be in line with our results. It is worth noting that the average PFS and OS of the patients in this study were 12.1 months and 15.5 months, respectively, which remains various from the results obtained in the above prospective study. The difference in survival outcomes may be explained by the bias brought about by highly selective patients. In summary, our investigations provide evidence of clinical efficacy of the BR regimen for Chinese B-cell-associated iNHL patients.

Although extensive research has been carried out on treatment for specific NHL, few studies explore the impact of NHL subgroups on clinical efficacy. The clinical efficacy of the BR regimen is a controversial and much-disputed subject. In the first-line treatment of patients with FL grade 3A, R-CHOP is superior to the BR regimen [24]. While another study disclosed that BR has less toxicity than R-CHOP, which can remarkably decrease recurrence rate and prolong PFS [25]. A recent retrospective study [26] assessed the efficacy and safety of BR and chlorambucil (Chl)-R in untreated CLL patients. Compared with the BR regimen, the Chl-R regimen achieves similar ORR, PFS, time to retreatment (TTR), and OS, but as a result of heterogenicity and extraheterogenicity toxicities of bendamustine, the dose of the BR regimen is less than that of the Chl-R regimen. This result is consistent with our results. Previous research discussed the clinical efficacy of various lymphomas. Moreover, our research included patients with different subgroups, and some patients had received antitumor therapy previously. Nonetheless, our research failed to unveil the impact of multiline treatment on the survival of patients.

Besides, multivariate Cox regression analysis disclosed that subtype was a factor that affected prognosis. But *β*2-MG levels before and after treatment are unable to predict a patient's prognosis well. The reasons may be related to multiplex subtypes and multiline treatment regimens. On the other hand, the results vary in different studies concerning the optimal critical value of *β*2-MG as a predictor [27], which may be due to distinct test methods. Considerably more work will need to be done on this issue.

This study was subjected to certain limitations. First, it was a retrospective study with a relatively low level of evidence. Besides, it was a single-arm study that could not be compared with current research programme. Second, this study was limited by small sample size, especially in various histological subtypes of B-cell-associated iNHL. A study [28] unraveled that BR has favorable clinical efficacy as a first-line treatment in unfit patients without TP53 disruption. Nevertheless, this study was limited by a lack of information such as gene mutations in patients. Third, the optimal dose of the BR regimen needs to be warranted. Finally, short follow-up time led to inaccuracy in judging survival of patients after BR regimen.

To put it succinctly, this study authenticated that the BR regimen had favorable efficacy and safety in patients with B-cell-associated iNHL. Though the *β*2-MG level did not play a prognostic role in this study, its potential value will be further determined in future studies. Overall, the findings of this study have a number of pivotal implications for future practice of the BR regimen for Chinese patients. Further research in clinical is, therefore, an essential next step in ascertaining the optimal therapeutic regimen.

## Figures and Tables

**Figure 1:** Survival curves: (a) PFS; (b) OS.

**Figure 2:** Comparisons of *β*2-MG level in two efficacy groups: (a) CR+PR vs. SD+PD before treatment; (b) CR+PR vs. SD+PD after treatment.

**Figure 3:** *β*2-MG level changes in the same group before and after treatment: (a) CR+PR before treatment vs. CR+PR after treatment; (b) SD+PD before treatment vs. SD+PD after treatment.

**Figure 4:** Subgroup survival curves of patients before treatment: (a) PFS of the *β*2‐MG < 3.25 mg/L group (blue) and the *β*2‐MG ≥ 3.25 mg/L group (red); (b) OS of the *β*2‐MG < 3.25 mg/L group and the *β*2‐MG ≥ 3.25 mg/L group.

**Figure 5:** Subgroup survival curves of patients after treatment: (a) PFS of the *β*2‐MG < 2.77 mg/L group (blue) and the *β*2‐MG ≥ 2.77 mg/L group (red); (b) OS of the *β*2‐MG < 2.77 mg/L group and the *β*2‐MG ≥ 2.77 mg/L group.

**Figure 6:** Subgroup survival curves of the *β*2-MG expression change rate: (a) PFS of the change rate < 0 group (blue) and the change rate > 0 group (red); (b) OS of the change rate < 0 group and the change rate > 0 group.

**Table 1:** Baseline characteristics of patients.

Characteristics	All patients, *N* = 73 (%)
Median age, years (IQR)	62 (56–69)
Sex, *n* (%)	
Male	41 (56.2)
Female	32 (43.8)
Histology, *n* (%)	
Mantle-cell lymphoma	17 (23.3)
Follicular lymphoma	20 (27.4)
Lymphocytic lymphoma (SLL/CLL)	11 (15.1)
Mucosa-associated lymphoid tissue	18 (24.7)
Other	7 (9.6)
Stage, *n* (%)	
I-II	13 (17.8)
III-IV	60 (82.2)
Prognostic groups for all patients (IPI), *n* (%)	
>2 risk factors	11 (15.1)
MIPI risk, *n* (%)	
Low (≤3)	4 (5.5)
Intermediate (4–5)	9 (12.3)
High (>5)	4 (5.5)
FLIPI risk, *n* (%)	
Low (≤1)	5 (6.8)
Intermediate (2)	3 (4.1)
High (3–5)	12 (16.4)
ECOG performance status	
0~1	59 (80.8)
≥2	14 (19.2)
Number of previous treatments	
1	33 (45.2)
≥2	40 (54.8)
Prior chemotherapy, *n* (%)	37 (50.7)
Previous rituximab treatment, *n* (%)	31 (42.5)
*β*2-MG (mg/L)	3.25 (2.28-4.89)

Abbreviations: IPI = International Prognostic Index; MIPI = mantle cell lymphoma IPI; FLIPI = follicular lymphoma IPI.

**Table 2:** Clinical efficacy.

Response (*n* = 73)	*n* (%)
ORR	58 (79.5)
CR	27 (37.0)
PR	31 (42.5)
SD	12 (16.4)
PD	3 (4.1)
Median PFS (95%CI)	12.1 (10.9-13.2)
Median OS (95%CI)	15.5 (14.8-16.1)

**Table 3:** Multivariate Cox regression analysis.

Variable	PFS		OS	
	HR (95%CI)	p value	HR (95%CI)	p value
Sex (female vs. male)				
Age (≤60 vs. >60)				
Type (B-cell associated indolent lymphoma vs. Mantle cell lymphoma)	2.645 (0.995-7.026)	0.051		
Stage (I-II stage vs. III-IV stage)				
ECOG PS (0-1 vs. ≥2)				
Number of treatment lines (first-line vs. ≥second-line or later)				
*β*2-MG (>3.5 mg/L vs. ≤3.5 mg/L)				

OS. HR (95%CI). *p* value.

**Table 4:** All-grade AEs.

Toxicities during BR	Major AEs^∗^ (%)	Grade 3-4 AEs (%)
Nausea and emesis	3 (4.1)	1 (1.4)
Leukopenia	6 (8.2)	5 (6.8)
Fatigue	4 (5.5)	
Infections	4 (5.5)	
Fever	3 (4.1)	
Rash	1 (1.4)	

∗: Major AEs include any grade of adverse events.

## Data Availability

The data used to support the findings of this study are included within the article. The data and materials in the current study are available from the corresponding author on reasonable request.
